# Assessing Physiochemical Characteristics of Agricultural Waste and Ready Compost at Wadi Al-Far'a Watershed of Palestine

**DOI:** 10.1155/2023/6147506

**Published:** 2023-01-30

**Authors:** Issam A. Al-Khatib, Fathi M. Anayah, Majed I. Al-Sari, Suha Al-Madbouh, Jumana I. Salahat, Baraa Y. A. Jararaa

**Affiliations:** ^1^Institute of Environmental and Water Studies, Birzeit University, P.O. Box 14, Birzeit, State of Palestine; ^2^College of Engineering and Technology, Palestine Technical University—Kadoorie, P.O. Box 7, Tulkarm, State of Palestine; ^3^Universal Institute of Applied and Health Research, Nablus, State of Palestine; ^4^The Joint Service Council for Solid Waste Management for Hebron and Bethlehem Governorates, Hebron, State of Palestine; ^5^Institute for Technology and Resources Management in the Tropics and Subtropics, TH Köln-University of Applied Sciences, BetzdorferStraße 2, 50679 Köln, Germany

## Abstract

The Wadi Al-Far'a Watershed (WFW) is one of the most important agricultural lands in Palestine where considerable amounts of organic wastes are generated. Yet, mismanagement of agricultural waste, including random disposal and/or burning, is a prevalent practice in the WFW. Such a practice might result in greenhouse gas emissions and leachate penetration into underlying soil and groundwater. To encourage compost production in the WFW as an efficient way for organic agricultural waste treatment and emission reduction, this study aims at evaluating the quality of both raw organic agricultural waste and ready compost, locally produced or imported. The evaluation considers the physiochemical characteristics as well as the heavy metal contents. The analysis of 17 samples of raw organic agricultural waste showed a good potential for compost production due to the high content of organic matter and other nutrients such as nitrogen and phosphorus. The analysis of 15 ready compost samples, however, showed that compost quality is relatively low due to the high electrical conductivity and low moisture content measurements as well as the high levels of sodium, chloride, and potassium. Furthermore, heavy metal contents of both raw organic agricultural waste and ready compost samples are less than the limits specified by the Palestinian and international standards. Therefore, local farmers can safely use raw organic agricultural waste generated in the WFW for compost production. Composting will not only enhance soil reclamation and crop production but also protect human health and the environment and promote sustainable economic development.

## 1. Introduction

Agricultural activities can generate considerable amounts and variety of organic wastes such as crop refuse, fruit and vegetable refuse, tree trimming waste, animal manure, and poultry manure. Organic waste can be a major threat to the environment, e.g., air pollution, if not managed and treated properly [1]. When landfilled, organic waste undergoes biological degradation process releasing methane gas (CH_4_), carbon dioxide (CO_2_), hydrogen sulfide (H_2_S), nitrous oxide (N_2_O), and other gases in small amounts [2, 3]. These gases are major contributors to the global warming and climate change as well [4].

Therefore, the European Union Landfill Directive (Directive 1999/31/EC) requires diverting organic waste sent to landfills in order to reduce the emission of greenhouse gases [5]. As indicated by the European Union Waste Framework Directive (Directive 2008/98/EC), final disposal or landfilling of waste becomes the least favorable option, and as a result, other sustainable management options such as recycling or composting are strongly advisable in the waste hierarchy [6–8].

Composting is considered one of the most efficient ways for organic waste treatment and emission reduction [9–11]. It has been recognized as an effective process for the treatment of animal manure [12–16], sludge [17, 18], and municipal solid waste [1, 6, 14, 19–21]. Composting domestic waste at household level can also promote a reduction in the emission of CH_4_ and N_2_O during decomposition and waste transformation [1, 2].

Composting agricultural and other types of organic wastes can be a useful process for recycling nutrients and maintaining organic matter in the soil when the end product of compost is used as a fertilizer or soil conditioner [8, 22, 23]. Composting can also reduce carbon to nitrogen (C/N) ratio of the organic waste to levels that are beneficial to the plants [23, 24]. Furthermore, composting can mitigate negative impacts such as plant pathogens and weed seeds [15, 25].

Farm waste composting is considered a resource for sustainable agriculture and plays an important role in organic farming practices. That is, it can reduce the use of chemical fertilizers and encourage compost application as an organic fertilizer that improves soil fertility [7, 25]. Application of organic amendments, coming from the composting process of different kinds of wastes, to the soil results in a significant improvement in the nutritional condition of plants as well as the growth and quality of harvested fruits [25–35].

The production of compost from organic refuse and its use in agricultural activities have been issues of interest by several studies [36–41]. However, the physiochemical characteristics and mixing ratios of raw organic waste, being the feedstock for compost production, need to be assessed [38, 42]. This is because the quality and portion of the feedstock used are the primary determinants of the composition and quality of the final compost, including its physiochemical properties [6, 43] and its maturation time [1, 39].

For instance, C/N ratios in the range of 25–40 can optimize the time needed for compost production, as these ratios accelerate the microbial activity and organic matter degradation and can result in good quality compost [39, 44]. Each type of organic waste contains a certain C/N ratio that differs from other types [24]. Therefore, the portion of each fraction is important to achieve the optimal C/N ratio at the beginning of the process in the range of 25–40 [23].

As for heavy metals, their presence in compost can reduce the quality of compost and create health risks if these metals exceed the limits specified by technical standard specifications [38, 45]. Heavy metals can enter the food chain through the plants, and their accumulation in the human body can create health risks and lead to death [46–48].

In the West Bank of Palestine, a recent study conducted in Hebron city by Al-Sari et al. [49] revealed that compost in the Palestinian markets is of medium quality due to partial or non-compliance with the quality standards and guidelines. This study showed that almost all Palestinian farmers are willing to use compost in their farms. The physical, chemical, and biological properties of the soil control its quality [6]. Contamination of agricultural soils has become a serious threat to food security and water resources in developing countries [50]. The effect of chemical fertilizers on four physiochemical properties and concentrations of seven heavy metals in agricultural soils of Libya was evaluated by Salem et al. [50]. While seasonal variation of physiochemical characteristics in agricultural soil was noticed because of agricultural activities, seven heavy metals of major concern were all below permissible limits.

In Iraq, five physiochemical parameters and two heavy metals in nine mixed samples of municipal solid waste with organic waste from different animal and plant sources were evaluated and found to be within the acceptable limits [8]. Kabasiita et al. [51] assessed the quality and fertility of municipal solid waste compost produced from 12 compost plants in Uganda. They assessed 10 physiochemical parameters and eight heave metals and found that the 12 compost plants produced low-fertility and poor-quality compost materials that did not meet several standards. In summary, adding organic additives to municipal solid waste is a key solution to improve the physiochemical characteristics of compost materials [8, 21].

However, studies assessing characteristics of compost feedstock and quality of ready compost used in agriculture are scarce in Palestine. Accordingly, the present research aims, first, to assess the physiochemical characteristics and heavy metal constituents of raw organic agricultural waste produced in the Wadi Al-Far'a Watershed (WFW) of Palestine, as a resource for farm composting. Secondly, the present study assesses the quality of ready compost available in the WFW for agricultural use including locally produced and imported compost.

## 2. Research Methods

### 2.1. Sampling

The WFW is one of the most important agricultural lands in the West Bank due to availability of fresh water resources for agricultural purposes, climatic variability, and high soil fertility. The WFW has an area of 331,000 dunums (1 dunum = 1,000 m^2^), constituting 6% of the West Bank area [52], which is inhabited by 60,927 people [53]. Its total agricultural area is 124,790 dunums, which constitutes 37.7% of the total land use in the WFW [52]. Growing fruits and vegetables and raising livestock are common agricultural activities in the WFW that can generate considerable amounts of organic waste. This waste stream is of much concern to both competent authorities and local farmers due to its possible health and environmental threats, particularly groundwater contamination, if not managed properly.

A total of 32 samples, including 17 samples of raw organic agricultural waste and 15 samples of ready compost, were randomly collected during September 2017. Different types of samples were collected from the following agricultural villages (Figure 1): 2 samples from Al-Bathan, 7 samples from Al-Far'a, 2 samples from An-Nassariya, 9 samples from Tammun, 8 samples from Talluza, and 4 samples of unspecified locations in the WFW. The collected raw organic agricultural waste was either freshly generated or old accumulated and piled without any further treatment. The raw organic agricultural waste included livestock (i.e., cow, sheep, and goat) manure, poultry manure, fruit residues, vegetable residues including leaves and branches, field crop (i.e., wheat, corn, and fodder) residues, and grass (Table 1). Ready compost samples were selected from locally produced and imported compost (Table 1).

### 2.2. Data Analysis

This research focuses on the quality parameters of raw organic agricultural waste and ready compost through laboratory testing. All of the collected samples were treated and tested in accordance with the standard procedures at the laboratories of the Palestinian National Agricultural Research Center located in Qabatiya of Jenin district. Laboratory testing was conducted for all samples considering the physical, chemical, and heavy metal parameters. The physiochemical parameters included electrical conductivity (EC), pH, nitrogen (N), phosphorous (P), potassium (K), sodium (Na), chloride (Cl), calcium (Ca), magnesium (Mg), moisture content (MC), organic matter (OM), and carbon to nitrogen ratio (C/N). The heavy metal parameters of concern included zinc (Zn), manganese (Mn), iron (Fe), chromium (Cr), cadmium (Cd), and lead (Pb).

It is worth to mention how these physiochemical and heavy metal parameters were measured in brief. First of all, the samples were analyzed in duplicate for a better analysis of the results. The minimum, maximum, average, and standard deviation values were used to describe the characteristics of the samples. In effect, a conductivity meter (AP-2, HM Digital, USA) detected the EC and a pH meter (PB-10, Sartorius, Germany) measured the pH [6, 50]; (Qiu et al., 2021). The wet samples were put in an oven at 90–105°C for 1-2 days to determine the dry weight and calculate the MC [21, 54]; (Qiu et al., 2021). The an EA1108 elemental analyzer equipped with an autosampler was used to compute the N, C, and OM contents of the samples [6, 21, 54]. In particular, the N value was determined by flame atomic absorption spectrometry [21, 46, 47, 50] following steam distillation and titration method [19].

The spectrophotometer analysis was used to determine the P content in compost samples digested in acid mixture [6, 8, 21, 55]; however, K was measured by a flame photometer [8, 19, 46, 47]. The procedure illustrated in the 3051A method of the United States Environmental Protection Agency [56] was adopted to determine the Na, Ca, and Mg contents of the samples. The saturated extract method was suitable to determine the Cl content of the compost samples [25].

As for the heavy metals, a quantitative analysis was performed according to the 3051A method of the US EPA [56]. The samples were dried, ground, and heated with nitric acid to determine the content of heavy metals using an inductively coupled plasma mass spectrometer [6, 54, 56]. In order to analyze the heavy metal contents (namely, Zn, Mn, Fe, Cr, Cd, and Pb), samples were burned in a silica crucible and digested in a Teflon beaker [6, 19, 57, 58]. Flame atomic absorption spectroscopy was used to compute Zn, Fe, and Mn concentrations of the samples, while Cd and Cr contents were calculated using mass spectrometry [8, 46–48, 57]. The polarographic analyzer using the square wave voltametric technique was used to analyze the Pb samples [8, 58].

## 3. Results and Discussion

### 3.1. Physiochemical Properties of Raw Organic Agricultural Waste

The characteristics of the raw organic agricultural waste play an important role in determining the quality of the compost produced from these materials. Studying the raw material contents can assist in estimating the portion of feedstock in the compost mixture to produce quality compost that complies with the standards. This study examines the physiochemical properties and heavy metal contents of the raw organic agricultural waste produced in the WFW as a resource for compost production in the area of study.  Table 2 presents the statistics of the tested physiochemical parameters to the 17 raw organic agricultural waste samples. The statistics include the minimum (Min), average, standard deviation (St. Dev.), and maximum (Max) values for each parameter of interest. For more illustration, the results found in Table 2 are explained as follows.

#### 3.1.1. Electrical Conductivity (EC)

The EC indicates the concentration of salts in the raw organic material. The EC of all tested samples was found in the range of 1.26–10.70 dS/m (deciSiemens per meter) with an average value of 6.10 dS/m (Table 2). None of the 17 samples exceeded the EC Jordanian standard for compost production of 15 dS/m as indicated by Al-Sari et al. [49]. Yet, 12 out of the 17 samples exceeded the World Health Organization (WHO) standard of 2–5 dS/m as specified by Azim et al. [59]. The average EC value was slightly higher than the optimum range of 2 to 4 dS/m for composting [60]. Yet, mixing different organic materials can reduce the high value of EC for some waste fractions. It was noticed that raw materials of fruit residues (i.e., W7 and W8) had the lowest EC values among all samples. In comparison to other studies in the Middle East region, EC was found to be 5.86 dS/m, on average, for several tested samples of compostable materials from Morocco as reported by Azim et al. [59]. As for the nine samples of Ajaweed et al. [8] taken from Iraq, EC ranged from 3.67 to 4.66 dS/m and agreed with the Jordanian [49] and WHO [59] standards. As for the 12 compost samples from Uganda [51], none of the samples violated the Jordanian standard, yet four samples only violated the WHO standard.

#### 3.1.2. pH

The pH values for all tested samples were in the range of 3.56–7.58 with an average value of 6.21 (Table 2), which was quite suitable for composting. For optimum growing media, pH should vary from 5.2 to 7.3 [61]. It was obvious that the raw materials of fruit residues (i.e., W7 and W8) had the lowest pH values compared to the other 15 samples. These two samples were the only ones that violated the Palestinian standard of 5.0–8.5 specified by Al-Sari et al. [49]. One of the 17 samples slightly exceeded the pH Jordanian standard for compost production of 7.5 [49]. Yet, only 6 samples were lower than the WHO standard of pH values in the range of 6–9 [59]. Previous studies reported that raw feedstock having a pH value within the range of 3–11 can also be composted [62, 63]. Compared to the Azim et al. [59] study in Morocco, the average pH value for samples of compostable materials was as high as 9.40. The pH values in nine samples of raw and mixtures of compost materials in Iraq were within the acceptable limits [8]. A total of 11 out of the 12 compost samples of Kabasiita et al. [51] from Uganda exceeded the Palestinian pH standard.

#### 3.1.3. Nitrogen (N)

All tested samples contained N in the range of 0.22–19.05% with an average value of 4.53%. Excluding the two samples of the poultry manure raw material (i.e., W4 and W11) with extreme values, the average and maximum values of N went down to 2.6 and 5.2%, respectively. The large variation in the N constituent could be attributed to the composition of the sample and the age of the material at the sampling time as N was reduced with time elapsed. The Jordanian standard [49] shows that the total N for compost production has to be ≥1.5%, while it is between 0.1 and 1.8% according to the WHO standard [59]. Three samples, namely W1, W7, and W13, were below the Jordanian standard (Table 2). Azim et al. [59] found the average total N content in raw organic agricultural waste for several tested samples from Morocco to be 0.87%. Azim et al. [59] reported the micronutrient contents (% weight/weight or w/w dry matter of N) as follows: citrus (0.69%), tomato (0.70%), banana (1.17%), sheep manure (1.19%), and other vegetable crops except tomato (2.38%). As for the 12 compost samples from Uganda [51], the N content varied between 0.3 and 0.6% which agreed with the WHO standard in contrast to the Jordanian one.

#### 3.1.4. Phosphorous (P)

The P content was relatively low and in the range of 0.01–0.17% with an average of 0.11%. It can be noticed that raw materials of fruit residues (i.e., W7 and W8) had the lowest P values compared to the other waste samples. However, the grass raw material (W16) had the highest values of *P* and pH but the lowest MC (Table 2). Azim et al. [59] also found that the P_2_O_5_ average value of several tested samples of raw organic wastes was 2.5%. The value of *P* as P_2_O_5_ should be from 0.10 to 2.30% for compost production according to the WHO standard [59]. Azim et al. [59] reported the micronutrient contents (% w/w dry matter of P oxide, P_2_O_5_) as follows: citrus (1.05%), tomato (0.31%), banana (0.31%), sheep manure (0.31%), and other vegetable crops except tomato (0.12%). As for the 12 compost samples from Uganda [51], the content of *P* ranged from 0.2 to 0.8% which agreed with the WHO standard.

#### 3.1.5. Potassium (K)

The content of K in all tested samples was in the range of 0.70–4.50% with an average of 1.68%. The maximum value of K was noticed for the poultry manure at Al-Far'a village, namely, W10 (Table 2). However, there are no limitations on the K content in the compost according to the Palestinian and Jordanian standards [49]. The WHO standard indicates that the value of K as K oxide, K_2_O, must be between 0.10 and 1.70% [59]. Azim et al. [59], however, found that the average value of K_2_O for several tested samples of raw organic wastes was 1.74%. Azim et al. [59] reported the micronutrient contents (% w/w dry matter of K oxide, K_2_O) as follows: citrus (0.95%), banana (1.8%), sheep manure (1.11%), and other vegetable crops except tomato (0.5%). As for the 12 compost samples of Kabasiita et al. [51] from Uganda, the K content varied from 0.7 to 2.3% with an average value of 1.3%, and only three samples exceeded the WHO standard.

#### 3.1.6. Sodium (Na)

All tested samples contained Na in the range of 0.02–0.25% with an average of 0.11%. As depicted in Table 2, fruit residues had the lowest Na values (i.e., W7 and W8), in addition to another sample of vegetable residues, namely, W14. The highest Na content was detected in the grass sample of W17. There are no specific limits for the Na contents in the compost according to the Palestinian, Jordanian [49], and WHO [59] standards. Azim et al. [59] found that the average value of Na as Na oxide (i.e., Na_2_O) for several tested samples of agricultural waste was 0.44%.

#### 3.1.7. Chloride (Cl)

The Cl parameter is not specified by the Palestinian and Jordanian compost standards [49]. However, the Cl content in all tested samples was in the range of 0.01–4.89% and the average value was 1.12% (Table 2). The fruit residue (W8) and the poultry manure (W4) samples had the minimum and maximum Cl contents, respectively.

#### 3.1.8. Calcium (Ca) and Magnesium (Mg)

As depicted in Table 2, the contents of Ca and Mg in all tested samples were in the range of 0.09–1.2% and 0.04–0.76%, respectively. The average values of Ca and Mg were 0.52 and 0.22%, respectively. The fruit residue (W8) and the poultry manure (W10) samples had the minimum and maximum Ca contents, respectively. All samples of livestock manure (i.e., W5 and W6) and fruit residues (i.e., W7 and W8) shared the lowest Mg content. Both parameters are not specified by the Palestinian and Jordanian compost standards [49]. The average values of CaO and MgO for several samples of raw organic waste from Morocco were found to be 6.78 and 0.79%, respectively [59]. It was noticed that the contents of Ca and Mg in the 12 compost samples from Uganda were in the range of 0.7–3.2% and 0.3–0.9%, respectively [51].

#### 3.1.9. Moisture Content (MC)

The MC of the 17 tested samples was in the range of 5.37–85.50%, and the average value was 19.61%. The optimum MC in the compost mixture shall be in the range of 40–60% [21, 23]. Other references in the literature showed a wider range of MC (i.e., 25–80%) for effective composting of organic materials [21]. This parameter can be easily controlled by water addition in case the MC is less than the required range or dewatering by adding dry matter when the MC is more than that range. Previous studies showed that the average value of MC for several samples of raw organic wastes was 36% [59].

#### 3.1.10. Organic Matter (OM)

Almost all raw organic samples contained good portion of OM which was in the range of 14.48–82.56%, and the average value was 66.82%. Matured compost shall contain OM not less than 25% based on the Palestinian standard, while the Jordanian standard shows that OM for compost production has to be ≥60% [49]. Only the two samples of fruit residue raw material (i.e., W7 and W8) were below the thresholds of the two standards (Table 2). Excluding these two extreme samples, the minimum and maximum values of OM boosted up to 63.47 and 82.56%, respectively. Elevated values of OM were noticed for all samples of field crop residues. Azim et al. [59] found that the average organic carbon content of several samples of raw organic wastes was 67.01%. While none of the nine samples of Ajaweed et al. [8] in Iraq exceeded the Palestinian standard, only five samples agreed with the Jordanian standard. It was shown that OM in the 12 compost samples from Uganda ranged between 7.8 and 28.6% with an average value of 15.2% [51]. While none of the 12 compost samples met the OM Jordanian standard, only one sample met the Palestinian standard.

#### 3.1.11. Carbon to Nitrogen (C/N) Ratio

All of the tested samples showed C/N ratios in the range between 2.00 and 59.90 with an average value of 18.09 (Table 2). The poultry manure (W11) and the field crop residue (W1) samples had the minimum and maximum C/N ratios, respectively. The variability in the ratio of C/N mainly depends on the original constituents as well as the age of the collected samples [1]. That is, the C/N ratio decreases as the material biologically degrades. Initial C/N ratios between 25 and 50 are optimal for aerobic composting [64, 65]. The Jordanian standard indicates that the C/N ratio for a stable compost production is almost ≤15, while the standard in the States is a C/N ratio of up to 25 [49]. It was obvious from Table 2 that only three samples of raw organic waste exceeded the C/N threshold of 25. Azim et al. [59] found that the average ratio of C/N of several samples of raw organic wastes was 39.79. Malakahmad et al. [63] reported C/N ratios of 9.26 and 61.32 for food waste and yard waste, respectively. It was found that only three out of the nine samples of Ajaweed et al. [8] from Iraq did not exceed the 25 ratio limit. As for the 12 compost samples of Kabasiita et al. [51] from Uganda, the C/N ratios ranged from 10.5 to 26.3 with an average value of 17.2, and only one sample violated the standard in the States.

### 3.2. Heavy Metal Contents of Raw Organic Materials

Heavy metals are characterized by high toxicity and can cause severe damage to the human health if they enter the food chain [6, 46–48, 50]. Therefore, the heavy metal concentration in organic fertilizers shall be within the limits specified by the Palestinian standard. Toxicity depends on the raw waste due to the presence of persistent organic pollutants or heavy metals [50, 66, 67] as well as the soil properties [6]. Hence, the parameters of heavy metal contents were tested for all collected raw waste samples.

The test results showed low concentrations of heavy metals that were considerably below the limits of the Palestinian standard. There is no surprise since it is well known that agricultural waste usually contains low levels of heavy metals [50, 61].  Table 3 presents the heavy metal contents of raw organic agricultural waste sampled from the WFW. It was noticed that the two samples of fruit residues (i.e., W7 and W8) had no contents of heavy metals at all.

The African Organization for Standardization had set the following limits (all in mg/kg) for heavy metals in compost materials: 40–100 for Zn, 200–800 for Mn, 1000–2500 for Fe, up to 50 for Cr, up to 5 for Cd, and up to 30 for Pb [51]. As for the 12 compost samples of Kabasiita et al. [51] from Uganda, violations to the African standard limits were recognized for the Zn, Fe, and Pb contents. None of the samples of the present study exceeded the African standard limits for the six heavy metals as depicted in Table 3. However, it would be interesting to discuss possible sources of these metals in solid waste.

Heavy metals might arise from domestic, agricultural, and industrial sources [68–70] and exist in raw organic agricultural waste with different levels of toxicity. Agricultural sources of heavy metals are pesticides, livestock manure, fertilizers, organic matter content, and wastewater [7, 50, 70, 71]. In effect, major sources of heavy metals include human excretion, galvanized materials, painting, mining, metallurgy, and corrosion of water supply and sewer systems [68, 71, 72].

At the household level, heavy metals may also come from kitchen cookware and sinks, dish washers, and washing machines. Some other applications involve high concentrations of heavy metals such as runoff from rooftops and use of laundry detergents and cleaning agents [69, 73]. Non-point sources of heavy metals include precipitation, weathering [72], road dust sediments [74], and traffic and combustion emissions [68]. In summary, heavy metals have been the sources of contamination to water, air, and land resources [19, 50, 72].

#### 3.2.1. Physiochemical Properties of Compost Samples

The physiochemical quality parameters for 15 compost samples were tested and compared to the limits specified in the Palestinian standard set by the Palestine Standards Institution (PSI).  Table 4 presents the results of these parameters in comparison with the national and international standards. Once a specific parameter is not specified by the PSI, it is compared with other international standard or guideline, e.g., the Jordan Standards and Metrology Organization (JSMO). All PSI and JSMO standards were specified by Al-Sari et al. [49]. Palestine and Jordan share the same physical and climatic conditions, and therefore, the comparison will be fair and justifiable. The WHO standard for compost production provided by Azim et al. [59] was also utilized for comparison purposes. The results are explained as follows.

*(1) Electrical Conductivity (EC)*. The EC of the 15 samples of ready compost varied from 3.47 to 8.88 dS/m with an average value of 6.22 dS/m (Table 4). Sample C6 was the only one that met the PSI limit of EC. None of the 15 samples exceeded the Jordanian standard of EC for compost production [49], yet 12 samples exceeded the WHO standard of 2–5 dS/m [59]. The average EC value was slightly higher than the optimum range of 2 to 4 dS/m for composting [60]. The average values of EC were too close for both the raw organic agricultural waste and the ready compost samples. Samples of ready compost produced by farmers (i.e., C5, C6, and C9) and locally produced (C13) had the lowest levels of EC. However, the highest EC measurements were observed in the ready compost samples produced by farmers (i.e., C3, C4, and C10) and imported (i.e., C1 and C2). In comparison to the previous study of Al-Sari et al. [49] for 14 ready compost samples from Palestine, the EC varied from 2.4 to 15.8 dS/m with an average value of 8.8 dS/m. Azim et al. [59], however, found that the average EC value for several samples of finished compost from Morocco was 3.77 dS/m. Khater [61] also found that the EC measurements for different compost types in Egypt ranged between 2.6 and 4.1 dS/m.

*(2) pH*. The pH values for all ready compost samples were in the range of 6.90–8.23 with an average value of 7.54 (Table 4). The minimum (C10) and the maximum (C5) values of pH were both of compost produced by farmers. All ready compost samples complied with the pH Palestinian specification [49] and consequently the WHO standard [59]. Almost seven of the 15 samples slightly exceeded the pH Jordanian standard for compost production. As for the 14 samples of ready compost found by Al-Sari et al. [49] in the Palestinian market, the pH varied between 6.56 and 8.88 with an average value of 7.60. As an example, the pH values for different compost materials from Egypt were in the range between 6.3 and 7.8 [61]. Compared to the Azim et al. [59] study in Morocco, the average pH value of finished compost samples from Morocco was 9.4.

*(3) Nitrogen (N)*. The N content in the ready compost samples ranged from 0.78 to 9.68% with an average value of 2.47% (Table 4). It was obvious that the maximum N value of 9.68% (C4 that is produced by farmers) is so extreme, and once it was excluded, the average and maximum N values would drop down to 1.96 and 4.66%, respectively. There is no specific limit provided by the PSI for the N content, the JSMO specifies its lower limit to be 1.5% [49], and it is between 0.1 and 1.8% according to the WHO standard [59]. Almost six and nine ready compost samples violated the JSMO and WHO standards, respectively. However, good quality compost should have a N content in the range of 0.4–3.5% [63, 75]. Accordingly, only two samples (i.e., C4 and C6) of compost produced by farmers exceeded the upper limit. As for the 14 samples of ready compost available in Palestine examined by Al-Sari et al. [49], the total N content ranged from 0.08 to 2.60% with an average value of 1.39%. These figures were close to those of the present study. Furthermore, Azim et al. [59] found the average total N content of compost samples from Morocco to be 1.33%. Khater [61], however, found that the total N values for different compost types in Egypt ranged between 0.95 and 1.68%.

*(4) Phosphorous (P)*. The P contents of the 15 ready compost samples were significantly low and in the range of 0.06–0.17% with an average of 0.12% (Table 4). There is no specific value provided by the PSI or JSMO [49]. Yet, good compost quality should have P contents in the range of 0.3–3.5% [63, 75], and noticeably, none of the samples in the present study was within this particular range. Al-Sari et al. [49] found that P as PO_4_ varied between 0.0 and 0.3% and averaged at 0.15% among 14 compost samples from Palestine. Khater [61] found that the total *P* values for different compost types in Egypt were in the range from 0.27 to 1.13%. Azim et al. [59] also found that the P_2_O_5_ average value of compost samples was 1.62%. The value of *P* as P_2_O_5_ should be from 0.1 to 2.3% for compost production according to the WHO standard [59].

*(5) Potassium (K)*. The contents of K in the 15 ready compost samples ranged from 0.70–6.40% with an average value of 2.52% (Table 4). Both the minimum (C4) and maximum (C3) values of K were of compost produced by farmers (Table 1). However, there are no limitations on the K content in the compost according to the Palestinian and Jordanian standards [49]. Compared to the 14 compost samples Al-Sari et al. [49] had taken from Palestine, K ranged between 0.06 and 1.8% at an average of 0.57%. The total *P* values for different compost types in Egypt varied from 0.27 to 2.11% [61]. The WHO standard [59] indicates that the value of K as K oxide, K_2_O, must be between 0.10–1.70%. Azim et al. [59], however, found that the average value of K_2_O for several tested samples of compost was 1.58%.

*(6) Sodium (Na)*. All 15 ready compost samples contained Na in the range of 0.06–0.80% with an average value of 0.27% (Table 4). The Na parameter is neither specified by the PSI, nor the JSMO, nor the WHO compost standards. If compared to the German standard of 0.05% Na as reported by WRAP [76], none of the samples met the standard. Compared to the 14 compost samples Al-Sari et al. [49] had taken from Palestine, Na ranged between 0.02 and 0.26% and averaged at 0.10%. Azim et al. [59] found that the average value of Na as Na_2_O for several compost samples from Morocco was 0.29%.

*(7) Chloride (Cl)*. The Cl contents in the 15 samples in the present study were in the range of 0.24–2.00%, and the average value was 0.98% (Table 4). Both the minimum (C6) and maximum (C3) values of K were of compost produced by farmers (Table 1). The Cl parameter is neither specified by the PSI nor the JSMO standards of compost production [49]. In reference to the German standard of WRAP [76], compost must have a Cl value of less than 0.10%, and accordingly, none of the 15 samples complied with this standard. In comparison to the previous study of Al-Sari et al. [49] in Palestine, the 14 compost samples had Cl values from 0.01 to 0.35% with an average value of 0.10%. The discrepancy between these figures and the results of the present study was evident.

*(8) Calcium (Ca) and Magnesium (Mg)*. As depicted in Table 4, the Ca and Mg contents in the 15 ready compost samples were in the range of 0.01–0.54% and 0.00–0.50%, respectively. The average values of Ca and Mg were 0.25 and 0.17%, respectively. The locally produced (C15) and the unspecified (C13) samples shared the minimum Ca and Mg contents. However, the compost produced by farmers had the maximum Ca (C10) and the maximum Mg (C7) values. Both parameters are not specified by the Palestinian and Jordanian compost standards [49]. In the previous study of Al-Sari et al. [49], the compost samples had Ca values from 0.00 to 0.60% with an average value of 0.08%. In the same study, the 14 compost samples had Mg levels between 0.00 and 0.13% averaged at 0.04%. The figures of Al-Sari et al. [49] were below those of the present study. This indicates how compost can be influenced by physical and climatic conditions as well as the other key parameters such as time elapsed, i.e., compost maturity and stability [1, 39, 77]. When compared to the study of Azim et al. [59] in Morocco, the average values of CaO and MgO for several compost samples were 5.30 and 0.81%, respectively.

*(9) Moisture Content (MC)*. The MC values of 14 ready compost samples (excluding C15) ranged from 4.01 to 38.61%, and the average value was 13.70% (Table 4). In fact, 6 out of the 14 MC samples in the present study exceeded the 12% standard of the JSMO [49]. The optimum MC in the compost mixture, however, shall be in the range of 40–60% [23], reflecting wet conditions. This contradiction between the compost standards indicates that the composition of compost significantly depends on its application and uses [77]. The MC considerably affects compost handling as dry compost of 35% MC or less is dusty while wet compost of more than 35% MC is heavy and clumpy [77]. Therefore, compost materials of MC of 30–60% are generally preferred for different applications [77], making only two samples of imported compost (i.e., C2 and C14) in the present study fell within the limits. Previous studies showed that the average value of MC for several compost samples from Morocco was 37% [59].

*(10) Organic Matter (OM)*. The measurements of OM varied from 22.00 to 75.40%, and the average value was 44.86% (Table 4). Matured compost shall contain OM more than 25% based on the Palestinian standard, while the Jordanian standard shows that the OM has to be at least 60% for compost production [49]. Again, the standards do not adopt the same threshold values, and this mainly depends on many factors of which the common application of compost is the key [19, 51, 77]. A total of four samples of compost produced by the farmers (i.e., C3, C4, C6, and C7) satisfied the JSMO standard; however, just three samples (i.e., C9, C11, and C14) violated the PSI standard (Table 4). For comparison purposes, a total of nine samples of ready compost in the present study complied with the USCC [77] guidelines that require OM in the range of 30–70%. When compared to the previous study of Al-Sari et al. [49] of 14 compost samples from Palestine, OM varied from 5.74 to 56.4% with an average value of 27.8%. Azim et al. [59] found that the average organic carbon content of several compost samples in Morocco was 63.25%. As for the results of the Khater [61] study in Egypt, the compost samples had OM values between 28.60 and 41.20%.

*(11) C/N Ratio*. The ready compost samples achieved C/N ratios in the range between 4.00 and 53.30%, and the average value was 14.62% (Table 4). During the composting process, C/N ratios within the range of 25 : 1 to 40 : 1 result in an efficient process while a C/N ratio of 30 is optimal [44]. A total of nine ready compost samples met the JSMO standard of the C/N ratio for stable compost production [49]. Only one sample of compost produced by farmers (C7) violated the standard of C/N ratio of 25 [6, 21] adopted in the States [49]. Excluding the extreme sample (C7), the average and maximum values of C/N ratio went down to 11.86 and 17.10, respectively. However, there is no specific value set by the PSI for the C/N ratio in the final compost [49]. In comparison with other standards, the matured compost shall have C/N ratio of less than 17 in California [78], less than 29 in Ethiopia, and less than 25 in Canada and Europe [21]. In the United Kingdom, the C/N ratio for final compost to be used for grass establishment shall not exceed 20 [78]. Compared to the standards, almost all ready compost samples of the present study, but not C7, met the required thresholds. It is worth to mention that none of the ready compost samples met the WHO standard of the C/N ratio which should be between 20 and 30 [59]. Al-Sari et al. [49] showed that the C/N ratio varied from 4.0 to 16.8 with an average value of 10.0. These figures strongly agree with the results of the present study, given that sample C7 is totally ignored. As for the study of Khater [61] in Egypt, the compost samples had C/N ratios between 14.22 and 18.52. Azim et al. [59] found the average C/N ratio for different compost samples from Morocco to be 23.92.

### 3.3. Heavy Metal Content of Compost Samples

Analyses of the heavy metal parameters of compost samples had been conducted by comparing local and international standards as depicted in Table 5. The Iranian and German standards indicated by Jalalipour et al. [79] were utilized for comparison purposes. Iran is a developing country which lies in the Middle East, while Germany is a European developed country in which environmental laws are stricter and limits are more stringent. The African standard [51], however, was surprisingly stricter than the German standard for the heavy metals except the Cd content (Table 5).

The results showed that the values of Zn, Cr, Cd, and Pb complied with the Palestinian, Iranian, German, and African standards. The only exception was the Cd values for 12 ready compost samples that exceeded the most stringent German standard of 1.00 mg/kg (or ppm), while only one sample, namely, C10, violated the African standard. The values of Mn and Fe are not specified in the Palestinian standards or any other international standards and guidelines [49, 79], except the African standard [51]. Table 5 displays the results of heavy metal contents of ready compost used in the WFW. With one exception (imported compost C2), almost all ready compost samples had higher values of Mn and Fe heavy metals compared to the contents of the other heavy metals. Noticeably, the compost sample produced by farmers (C8) had the lowest Fe and the second lowest Mn levels. With the exception of the Cr content, C9 had contents above the average corresponding values for other five heavy metals.

## 4. Conclusions and Recommendations

This study aims to assess the physiochemical characteristics of raw organic agricultural waste produced in the Wadi Al-Far'a Watershed (WFW) for the sake of potential compost production. It also evaluates the quality of the ready compost used by some farmers in the WFW, including locally produced and imported compost. To achieve the study objectives, 32 samples were selected from different agricultural villages in the study area. The samples consisted of 17 samples of raw organic agricultural waste and 15 samples of ready compost. Analysis of the physiochemical and heavy metal parameters of the raw organic agricultural waste revealed good potential for compost production due to its high content of organic matter and other nutrients such as nitrogen and phosphorous. However, the analysis of the compost samples showed that the compost quality was relatively low due to its high electrical conductivity, low moisture content measurements, and its high concentrations of sodium, chloride, and potassium.

More efforts are needed to improve compost quality in the local market. At the farming community level, there is a high potential to promote composting practices among farmers in the study area due to the good quality of raw materials. At the policy level, however, more efforts should be directed to improve the quality of compost, adopt proper guidelines and standards, raise awareness among farmers on how to produce and apply compost, and conduct effective training sessions to let farmers practice their knowledge and skills they acquire.

Composting has great impacts on economic development and environmental sustainability of agricultural communities. Local farmers at WFW are advised to reuse raw organic agricultural waste for composting which reduces both pollution and cost of fertilizers. Soil reclamation is to be enhanced by converting agricultural wastes into resources and returning nutrients needed for agricultural production. This is one of the principles of the circular economy to tackle global challenges such as climate change and waste management. Similar to other developing countries, Palestine has to develop a circular economy strategy that increases investment opportunities, prevents environmental degradation, and builds resilient communities [80].

## Figures and Tables

**Figure 1:** The agricultural villages of the Wadi Al-Far'a Watershed in Palestine.

**Table 1:** The description of the 17 raw organic agricultural waste (a) and the 15 ready compost (b) samples.

(a) The 17 raw organic agricultural waste samples				
Waste	Village			
	Al-Far'a	An-Nassariya	Tammun	Talluza
Livestock manure		W6		W5
Poultry manure	W10		W11	W4
Fruit residues	W8	W7		
Vegetable residues	W12, W14		W9, W13	
Field crop residues	W1			W2, W3
Grass	W15		W16, W17	

(b) The 15 ready compost samples				
Source	Sample Number			
Imported (ready)	C1, C2, C14			
Produced by farmers	C3, C4, C5, C6, C7, C8, C9, C10			
Locally produced (ready)	C11, C15			
Municipal waste	C12			
Unspecified	C13			

**Table 2:** Physiochemical properties of raw organic agricultural waste produced in the WFW.

Sample no.	EC (dS/m)	pH	N (%)	P (%)	K (%)	Na (%)	Cl (%)	MC (%)	OM (%)	Ca (%)	Mg (%)	C/N
W1	6.00	6.45	0.80	0.08	0.90	0.09	0.36	10.14	82.49	0.42	0.14	**59.90**
W2	6.40	6.67	1.95	0.13	1.00	0.08	0.44	9.44	**82.56**	0.61	0.22	24.60
W3	9.60	6.60	2.57	0.16	*0.70*	0.10	0.25	10.24	75.22	0.76	0.26	17.00
W4	5.63	6.88	**19.05**	0.13	1.00	0.12	**4.89**	10.15	77.18	0.37	0.09	2.30
W5	4.03	7.02	5.21	0.12	1.00	0.06	0.87	21.97	67.05	0.19	*0.04*	7.50
W6	5.66	7.03	2.84	0.15	1.60	0.08	0.96	23.03	66.05	0.10	*0.04*	13.50
W7	2.17	3.71	*0.22*	0.05	*0.70*	*0.02*	0.03	85.27	*14.48*	0.17	*0.04*	38.20
W8	*1.26*	*3.56*	4.07	*0.01*	1.40	0.02	*0.01*	**85.50**	14.50	*0.09*	*0.04*	2.10
W9	8.10	5.37	2.91	0.06	2.00	0.15	2.01	9.15	74.75	0.78	0.47	14.90
W10	4.65	6.97	2.60	0.16	**4.50**	0.08	0.69	5.72	72.59	**1.20**	0.54	16.20
W11	4.00	7.35	18.55	0.13	1.00	0.20	0.49	11.41	63.47	0.24	*0.04*	*2.00*
W12	8.90	5.47	3.21	0.12	2.80	0.10	1.45	8.95	78.76	0.73	0.25	14.20
W13	6.40	5.20	1.37	0.13	1.20	0.20	1.14	9.09	76.35	0.66	0.26	32.40
W14	10.70	6.90	3.71	0.07	1.20	*0.02*	2.00	10.66	67.84	1.00	**0.76**	10.60
W15	**6.10**	5.90	3.01	0.08	2.80	0.15	0.36	9.07	78.39	0.28	0.05	15.10
W16	6.21	**7.58**	3.22	**0.17**	2.40	0.15	1.38	*5.37*	70.86	0.65	0.21	12.80
W17	7.90	6.91	1.75	0.11	2.40	**0.25**	1.75	8.26	73.36	0.65	0.24	24.30
Min	1.26	3.56	0.22	0.01	0.70	0.02	0.01	5.37	14.48	0.09	0.04	2.00
Average	6.10	6.21	4.53	0.11	1.68	0.11	1.12	19.61	66.82	0.52	0.22	18.09
St. Dev.	2.48	1.19	5.50	0.04	1.02	0.07	1.17	25.20	20.44	0.32	0.21	14.70
Max	10.70	7.58	19.05	0.17	4.50	0.25	4.89	85.50	82.56	1.20	0.76	59.90

Minimum values are indicated in italics. Maximum values are indicated in bold.

**Table 3:** Heavy metal contents of raw organic agricultural waste produced in the WFW.

Sample no.	Heavy metal content (mg/kg)					
	Zn	Mn	Fe	Cr	Cd	Pb
W1	0.83	2.78	155.25	2.40	*0.00*	1.15
W2	1.20	414.50	114.53	0.10	*0.00*	*0.00*
W3	0.83	**440.35**	286.13	3.95	0.08	0.05
W4	1.08	292.55	249.28	2.80	*0.00*	2.05
W5	1.08	306.13	190.95	1.25	*0.00*	2.43
W6	1.13	305.63	37.08	**10.13**	3.68	0.23
W7	*0.00*	*0.00*	*0.00*	*0.00*	*0.00*	*0.00*
W8	*0.00*	*0.00*	*0.00*	*0.00*	*0.00*	*0.00*
W9	0.30	56.45	244.53	6.28	**3.73**	2.05
W10	0.70	85.40	248.90	6.65	2.60	**6.08**
W11	0.83	126.90	237.30	3.18	1.05	5.53
W12	0.53	310.08	213.45	3.18	1.28	4.25
W13	0.83	143.10	189.73	5.88	2.43	2.43
W14	0.55	136.30	189.30	4.33	0.60	3.70
W15	1.08	199.60	206.38	9.35	0.15	2.78
W16	**1.90**	249.30	183.23	6.65	0.30	4.63
W17	1.43	207.93	**299.50**	*0.00*	3.68	2.43
Min	*0.00*	*0.00*	*0.00*	*0.00*	*0.00*	*0.00*
Average	0.84	192.76	179.15	3.89	1.15	2.34
St. Dev.	0.48	140.04	91.78	3.21	1.46	1.98
Max	**1.90**	**440.35**	**299.50**	**10.13**	**3.73**	**6.08**

Minimum values are indicated in italics. Maximum values are indicated in bold.

**Table 4:** Physiochemical properties of compost used for agriculture in the WFW.

Sample no.	EC (dS/m)	pH	N (%)	P (%)	K (%)	Na (%)	Cl (%)	Ca (%)	Mg (%)	MC (%)	OM (%)	C/N ratio
C1	8.30	7.57	2.58	**0.17**	6.00	0.14	1.03	0.34	0.34	9.60	46.30	10.40
C2	7.61	8.21	2.67	0.14	2.25	0.15	0.55	0.35	0.11	37.21	38.03	8.30
C3	7.05	7.27	2.58	0.11	**6.40**	*0.06*	**2.00**	0.20	0.07	9.69	74.73	16.80
C4	**8.88**	7.21	**9.68**	0.15	*0.70*	0.28	1.87	0.19	0.05	10.95	67.03	*4.00*
C5	5.04	**8.23**	2.15	0.13	2.40	0.24	1.44	0.15	0.02	20.17	56.57	15.30
C6	*3.47*	7.08	4.66	0.16	1.00	0.12	*0.24*	0.20	0.05	10.68	**75.40**	9.40
C7	5.60	7.34	0.79	0.09	2.25	0.14	0.69	0.52	**0.50**	5.38	72.74	**53.30**
C8	6.97	7.77	2.07	*0.06*	1.80	0.14	1.42	0.36	0.22	6.91	38.75	10.90
C9	4.74	7.61	*0.78*	0.15	1.50	0.15	0.64	0.45	0.27	7.73	22.64	16.90
C10	7.60	*6.90*	1.61	0.13	2.00	0.20	1.10	**0.54**	0.36	7.21	31.75	11.40
C11	5.67	7.67	0.83	0.13	3.75	0.11	0.73	0.40	0.49	*4.01*	24.50	17.10
C12	6.70	7.46	1.25	0.07	1.40	**0.80**	1.11	0.02	0.01	6.89	33.96	15.70
C13	4.70	8.02	2.32	0.10	2.10	0.50	0.61	*0.01*	*0.00*	16.73	34.68	8.70
C14	5.50	7.46	1.15	0.10	1.80	0.60	0.62	0.02	0.01	**38.61**	*22.00*	11.10
C15	5.50	7.25	1.97	0.10	2.40	0.42	0.69	*0.01*	*0.00*		33.89	10.00
Min	*3.47*	*6.90*	*0.78*	*0.06*	*0.70*	*0.06*	*0.24*	*0.01*	*0.00*	*4.01*	*22.00*	*4.00*
Average	6.22	7.54	2.47	0.12	2.52	0.27	0.98	0.25	0.17	13.70	44.86	14.62
St. Dev.	1.51	0.39	2.23	0.03	1.65	0.21	0.51	0.19	0.18	11.12	19.39	11.35
Max	**8.88**	**8.23**	**9.68**	**0.17**	**6.40**	**0.80**	**2.00**	**0.54**	**0.50**	**38.61**	**75.40**	**53.30**
PSI	≤4	5–8.5								25–40	>25	
JSMO	≤15	≤7.5	≥1.5							≤12	≥60	≤15

Minimum values are indicated in italics. Maximum values are indicated in bold.

**Table 5:** Heavy metal contents of ready compost used for agriculture in the WFW.

Sample no	Heavy metal content (mg/kg)					
	Zn	Mn	Fe	Cr	Cd	Pb
C1	0.85	**433.90**	308.28	2.03	4.48	*0.00*
C2	0.98	*3.93*	283.60	**5.50**	1.00	5.18
C3	*0.00*	357.05	259.83	2.80	1.33	0.95
C4	0.83	318.73	273.95	3.95	1.68	0.23
C5	0.48	271.55	308.28	5.10	0.83	1.50
C6	1.55	362.25	234.53	2.03	0.20	4.08
C7	**2.08**	90.83	301.20	*0.00*	3.50	8.30
C8	1.13	15.25	*226.63*	*0.00*	1.50	7.38
C9	1.13	367.23	**332.60**	*0.00*	2.83	6.45
C10	*0.00*	68.98	314.23	*0.00*	**8.68**	8.68
C11	*0.00*	139.78	313.98	*0.00*	3.90	3.53
C12	*0.00*	276.70	327.00	*0.00*	3.98	11.43
C13	*0.00*	32.28	328.38	*0.00*	2.70	**18.13**
C14	*0.00*	45.73	313.45	*0.00*	1.95	8.48
C15	*0.00*	117.33	313.83	*0.00*	*0.00*	10.88
Min	*0.00*	*3.93*	*226.63*	*0.00*	*0.00*	*0.00*
Average	0.60	193.43	295.98	1.43	2.57	6.35
St. Dev.	0.68	151.70	33.27	2.02	2.19	4.96
Max	**2.08**	**433.90**	**332.60**	**5.50**	**8.68**	**18.13**
PSI	2500			400	20	300
Iranian standard	1300			150	10	200
German standard	300			70	1	100
African standard	100	800	2500	50	5	30

Minimum values are indicated in italics. Maximum values are indicated in bold.

## Data Availability

The datasets generated and/or analyzed during the current study are available from the corresponding author on reasonable request.
